The article "Effect of Repeated Firings and Thickness on Optical Properties of Variable Preshaded and Shaded Novel Translucent Zirconia Blocks" was published in 2022. Journal: Biomed Res Int.

# Effect of Repeated Firings and Thickness on Optical Properties of Variable Preshaded and Shaded Novel Translucent Zirconia Blocks

**DOI:** 10.1155/2022/8572782

**Published:** 2022-08-16

**Authors:** Bike Altan, Sevki Cinar

**Affiliations:** Department of Prosthodontics, Faculty of Dentistry, University of Health Sciences, Uskudar, Istanbul, Turkey

## Abstract

**Objective:**

The purpose of this study was to examine the optical properties of translucent zirconia with different thickness during multiple firings.

**Materials and Methods:**

Three different types of translucent zirconia (Vita YZ HT (HT), Vita YZ ST (ST), Vita YZ XT (XT)) with thickness of 0.5, 1, and 1.5 mm were used in the study. 180 disk-shaped specimens (*n* = 10) were prepared from preshaded and nonshaded blocks. The coloring liquid (A2, Vita Shade Liquid) was applied with a synthetic nylon brush in the nonshaded group. Then, the specimens were then subjected to 1, 3, and 5 firing times. After consecutive firings, color differences (Δ*E*) and translucency parameter (TP) were measured. Statistical analysis was carried out by using repeated measure ANOVA followed by Tukey test.

**Results:**

ANOVA analysis reveals that TP and Δ*E* were significantly affected by the repeated firings. The highest TP was seen in 0.5 mm XT specimen. For all specimens, TP decreases from 1st to 3rd firing cycles, despite TP increases from 3rd to 5th firing cycles. Although there is a significant change in TP values in 0.5 mm thickness, there is no significant change between firing cycles for 1 and 1.5 mm thickness specimens. The highest Δ*E* value was observed for shaded specimens between 1st and 5th firings. Δ*E* values were not significantly different between 1 and 3 firings.

**Conclusions:**

Changes in thickness and repeated firings of zirconia specimens affected final color and translucency of zirconia specimens. HT blocks are more affected by consecutive firings than ST and XT blocks. Δ*E* increased as the thicknesses decreased for both types of translucent zirconia specimens tested.

## 1. Introduction

In recent years, patient's demands for esthetic dentistry have increased. To achieve optimal esthetics and meet patients' request, it is essential for restoration to reach natural translucency of the teeth. Improved translucency of blanks and different coloring methods make it possible to produce restoration with natural tooth color and translucency [1].

Translucency of zirconia is mainly dependent on light scattering and thickness [2]. Also, yttria content, phase composition, grain size, number of firings, sintering temperature, and coloring method are crucial factors that affect the translucency and color of zirconia [3–5]. Translucency was determined by spectrophotometers which measure the spectral reflectance of an object one wavelength at a time and converts it into numerical form [6].

The article "Effect of Repeated Firings and Thickness on Optical Properties of Variable Preshaded and Shaded Novel Translucent Zirconia Blocks" was published in 2022. Journal: Biomed Res Int.

Translucent zirconia blanks are introduced to market as nonshaded (white) and preshaded. Preshaded blanks are more advantageous since they have more uniform color than nonshaded ones [7]. Coloring liquids are commonly used for compensating the white color of zirconia and also give restorations lifelike appearance and characterization [8, 9]. Final color depends on different pigment types and ratios in coloring liquids [10].

Restorations can be fired 2 to 5 times due to some shape and color corrections to satisfy esthetic demand of both patient and clinician. Besides, multiple firings are generally necessary after occlusal adjustments. Various studies have reported that firing causes color changes due to pigment breakdown during firing [11, 12]. O'Brien et al. [13] reported the perceivable color differences of specimens between 3rd and 5th firings. Firing processes can cause changes on optic and mechanical properties of the zirconia [14]. After repetitive firing procedures, differences in flexural strength, microhardness, and marginal fit can be seen in zirconia [15].

There is no study regarding repeated firings on optical properties of newly introduced extra- and high-translucent zirconia. Therefore, this study is aim at revealing if multiple firings can alter translucency and color of translucent zirconia. Additionally, this research is aimed at exploring which of the preshaded or shaded provide better optical properties after repeated firings. This research will enable us to see how the zirconia blanks are affected by the firing processes in terms of optical properties thus enabling dental practitioners to have an ideal approach in their clinical and laboratory practice.

The initial hypothesis is that repeated firings would not affect the translucency and color of high- and extratranslucent zirconia. The second hypothesis states that there is no significant color and translucency parameter (TP) change between preshaded and shaded blocks.

## 2. Materials and Methods

The composition, sintering conditions, and manufacturer of the materials used in this study are presented in Table 1. Three different types of translucent zirconia specimens (preshaded+nonshaded) were divided into 3 groups regarding the thickness (0.5, 1, and 1.5 mm). The study consists of 180 disk-shaped specimens (*n* = 10). These were fabricated from VITA YZ XT (XT), VITA YZ ST (ST), and VITA YZ HT (HT) (Vita Zahnfabrik, Germany) with the help of CAD/CAM system (Cerec inLab, Dentsply Sirona, York, PA). After milling, the coloring liquid (A2, VITA Shade Liquid XT, ST, HT) was applied with a synthetic nylon brush in the nonshaded group. Since most of the clinical color selection is from A2 color, this hue was selected. Then, excess water was wiped off and air-dried. Then, the specimens were predried in a drying cabinet for 15 min at 150 C. After drying process, Vita YZ HT (10 hours) and XT (7 hours) were sintered in firing furnace (Vita Zyrcomat 6000 MS) at 1450 C (4 hours 1530 C for Vita YZ ST) as per the manufacturer's recommendations. After sintering, thickness of specimens was checked with digital caliper (Mitutoyo Corp., Tokyo, Japan) with the accuracy of 0.01 mm.

The article "Effect of Repeated Firings and Thickness on Optical Properties of Variable Preshaded and Shaded Novel Translucent Zirconia Blocks" was published in 2022. Journal: Biomed Res Int.

After the specimens were ultrasonically cleaned in distilled water for 5 min, the translucency and color of the test specimens were evaluated using a spectrophotometer (VITA Easyshade V, VITA Zahnfabrik, Germany). Every specimen was subjected to repeated firings. Measurements were performed in first, third, and fifth firings by the same operator. Each value was recorded on five different areas of each specimen including the center of specimen [16].

CIE-Lab (Commission International de l'Eclairage *L*∗, *a*∗, *b*∗) values of each specimen were measured on a black background and on a white background with a spectrophotometer in the wavelength range of visible light, 400 to 700 nm, at 10 nm intervals. D65 illuminant and 2-degree observer were selected.

*L* represents the brightness of an object, *a* represents the red or green chroma, and the *b* represents the yellow or blue chroma. TP was obtained by calculating the color difference of the specimen over the black and white backgrounds with the following equation:

(1) $$\begin{array}{c} \text{TP}={\left[{\left(L_{b}*-L_{w}*\right)}^{2}+{\left(a_{b}*-a_{w}*\right)}^{2}+{\left(b_{b}*-b_{w}*\right)}^{2}\right]}^{1/2}. \end{array}$$

The color differences between firings were calculated for each specimen on software according to the formula: Δ*E*∗ = [(Δ*L*∗)^2^ + (Δ*a*∗)^2^ + (Δ*b*∗)^2^]^1/2^.

Statistical analyses were performed with the SPSS version 23.0 (IBM SPSS Statistics for Windows, v23.0; IBM Corp.). The conformity of the variables to the normal distribution was examined by histogram graphs and Kolmogorov-Smirnov/Shapiro-Wilk test. Mean and standard deviation values were used when presenting descriptive analyzes. ANOVA was performed for repeated measurements, taking into account the number of firings as repeated measurements and block and staining and sample thicknesses as intergroup factors. Considering the significant interaction effects between all factors, in one-sample repeated measurements, ANOVA and Sidak pairwise comparison tests were used to separately compare the mean values of light transmittance and the color change (Δ*E*) of different numbers of firings at each sample thickness and staining type. In addition, the mean values of different sample thicknesses for each firing number and staining type were compared using one-way ANOVA and the Tukey HSD test. The independent *t*-test was used to compare the mean values between the two staining types at each sample thickness and the number of individual firings. Cases with a *p* value below 0.05 were considered as statistically significant results.

The article "Effect of Repeated Firings and Thickness on Optical Properties of Variable Preshaded and Shaded Novel Translucent Zirconia Blocks" was published in 2022. Journal: Biomed Res Int.

## 3. Results

Repeated measure ANOVA analysis in Tables 2 and 3 reveals that TP and Δ*E* were significantly affected by the repeated firings.

Table 4 displays that TP decreases from 1st to 3rd firing cycle, despite TP increases from 3rd to 5th firing cycles for all specimens. Although there is a significant change in TP values in 0.5 mm thickness (*p* < 0.05), for 1 and 1.5 mm thickness specimens, there is no significant change between firing cycles (*p* > 0.05).

While the highest TP (27.63 ± 1.10) was seen in 0.5 mm XT specimen, the lowest TP (10.10 ± 0.46) was seen in 1.5 mm HT specimens. In addition, the TP values of the preshaded samples were found to be higher than the shaded samples. It was determined that the TP change was higher in shaded ones with repeated firings, but this change was significant only in 0.5 mm samples and insignificant in other thicknesses (1 and 1.5 mm).

According to Table 5, the highest Δ*E* value (7.05 ± 0.19) was observed for shaded specimens between 1st and 5th firings. Δ*E* values were not significantly different between 1 and 3 firings. Δ*E* values between 1st and 3rd and 3rd and 5th were below clinically perceivable threshold except between 1st and 5th firings which was above the threshold. Δ*E* change is higher in extra- and supertranslucent blocks than in translucent blocks.

As the thickness increases, Δ*E* values decrease. It was observed that Δ*E* change was more in thick samples after the first firing, whereas there was less change in Δ*E* values in later firings. It was seen that thin samples were more affected by Δ*E* changes between 3-5 and 3-7 firings.

## 4. Discussion

In this study, the initial hypothesis was rejected because different porcelain thickness and number of firing cycles affected the final color and translucency of extra- and high-translucent zirconia. As a result of the repetitive firings, preshaded and shaded exhibited different translucency and color changes; second hypothesis was also rejected.

There are several studies reported that repeated firings resulted in changes on optical properties of zirconia [17–19]. On the contrary, Ozdogan and Ozdemir's study [20] revealed that repetitive firings did not affect color and translucency of zirconia frameworks. Results of our study were in accordance with those of who reported repeated firing effect the color of zirconia.

The article "Effect of Repeated Firings and Thickness on Optical Properties of Variable Preshaded and Shaded Novel Translucent Zirconia Blocks" was published in 2022. Journal: Biomed Res Int.

The experimental results showed that thickness affected the translucency and color of monolithic zirconia which was consistent with previous studies [21, 22]. In the present study, translucency decreased when the thickness of materials increased which was in agreement with some studies [9, 21, 23].

The present study showed that thin specimens are more affected by repeated firings. The repeated firings changed the translucency 0.5 mm thick specimens but had no significant effect on 1 and 1.5 mm thick specimens. TP values are decreased from 1 to 3 firings, while translucency is increased from 3 to 5 firings for all thickness specimens which is consistent with conducted by Moon et al. [14] and Fathi et al. [18].

Using preshaded blocks and by staining white monolithic zirconia blocks in coloring liquids are two main approaches for coloring zirconia restorations [9, 24]. Coloring is essential to produce natural tooth-like restorations with a proper shade. In present study, preshaded blocks presented higher TP compared to shaded zirconia in each thickness group which is in agreement with Sen and Isler's study [25]. According to the results, preshaded blanks are more advantageous compared to nonshaded blanks since minor additional coloring is required to match the texture of natural adjacent teeth. Results of our study contradicts with Alp et al.'s study [26] which was found that externally shaded zirconia showed higher translucency than preshaded zirconia.

This study evaluated that shaded zirconia blocks showed higher color change according to preshaded zirconia. It may be attributed to preshaded zirconia color was homogeneous and more stable than nonshaded zirconia [16].

Based on the present study, the thickness of translucent zirconia influenced the Δ*E* values. Thicker specimens were less affected by repetitive firings according to thin specimens. 0.5 mm specimens were prone to color change after repeated firings while there is less color change in specimens with 1 and 1.5 mm thickness. This was consistent with the study of Fathi et al. [18] and Farzin et al. [27] which was reported that color change in thin specimens was more than thick specimens. Color change of thin specimens between firing cycles was above clinically acceptable threshold while color change with thicker veneers after repeated firings is below the threshold. 3.7 Δ*E* units were determined as a perceptibility threshold [13]. Dentists should consider when making thinner restorations, such as laminate veneers, that additional firings due to adjustments may result in color change and reduced translucency.

The article "Effect of Repeated Firings and Thickness on Optical Properties of Variable Preshaded and Shaded Novel Translucent Zirconia Blocks" was published in 2022. Journal: Biomed Res Int.

In the present study, while Δ*E* between 1 and 5 firings was significantly higher than that between 1 and 3 firings, Δ*E* between 3 and 5 firings was found least for all types of translucent zirconia blocks. Δ*E* between 1 and 5 firing cycles was above the clinically acceptable threshold (3.7 Δ*E*). These results were in accordance with those of Fathi et al. [18] who reported that Δ*E* between 1 and 3, 1 and 5, and 1 and 7 firings was significantly higher than that between 3 and 5, 3 and 7, and 5 and 7 firings.

Patients' esthetic demand is increasing for more and more translucent and natural restorations. It is essential to select most translucent type of block and appropriate shade and number of firings. It is crucial to minimize the influence of repeated firings which effect the final color and translucency of translucent zirconia. In choosing convenient materials, number of firing cycles and thickness of restoration should be considered.

## 5. Conclusions

Considering the limits of this investigation, the following conclusions were drawn: TP values of preshaded blocks were found higher than shaded blocks. Additionally, it was observed that Δ*E* increased as the thicknesses decreased for all types of translucent zirconia specimens tested. Since HT blocks were more affected by repetitive firings than ST and XT blocks, it can be recommended to be less preferred. Likewise, it should be taken into account that thin and shaded specimens were more affected by the multiple firings. Further studies are suggested to evaluate different types of restorations such as crowns and laminate veneers.

## Figures and Tables

**Table 1:** Chemical composition, sintering conditions, and manufacturer of materials.

Material	Composition	Sintering temperature/time	Manufacturer
VITA YZ XT (preshaded+nonshaded)	ZrO_2_ (86-91%) Y_2_O_3_ (8-10%) HfO_2_ (1-3%) Al_2_O_3_ (0-1%) Pigments (0-1%)	1450°C/7 hours	VITA Zahnfabrik, Germany
VITA YZ ST (preshaded+nonshaded)	ZrO_2_ (88-93%) Y_2_O_3_ (6-8%) HfO_2_ (1-3%) Al_2_O_3_ (0-1%) Pigments (0-1%)	1530°C/4 hours	VITA Zahnfabrik, Germany
VITA YZ HT (preshaded+nonshaded)	ZrO_2_ (90-95%) Y_2_O_3_ (4-6%) HfO_2_ (1-3%) Al_2_O_3_ (0-1%) Pigments (0-1%)	1450°C/10 hours	VITA Zahnfabrik, Germany

**Table 2:** Results of ANOVA for changes in color coordinates after repeated firings (TP).

Effect	Pillai value	*F*	Numerator df	Denominator df	Sig.
Number of firing	0.833	401.316	2	161	<0.001
Number of firing ^∗^ block type	0.086	3.646	4	324	0.006
Number of firing ^∗^ shade type	0.019	1.553	2	161	0.215
Number of firing ^∗^ thickness	0.157	6.904	4	324	<0.001
Number of firing ^∗^ block type ^∗^ shade type	0.144	6.292	4	324	<0.001
Number of firing ^∗^ block type ^∗^ thickness	0.171	3.796	8	324	<0.001
Number of firing ^∗^ shade type ^∗^ thickness	0.061	2.555	4	324	0.039
Number of firing^∗^ block type ^∗^ shade type ^∗^ thickness	0.071	1.497	8	324	0.157

ANOVA, *p* < 0.05 indicates a significant difference at repeated measurements.

The article "Effect of Repeated Firings and Thickness on Optical Properties of Variable Preshaded and Shaded Novel Translucent Zirconia Blocks" was published in 2022. Journal: Biomed Res Int.

**Table 3:** Results of ANOVA for changes in color coordinates after repeated firings (∆*E*).

Effect	Pillai value	*F*	Numerator df	Denominator df	Sig.
Number of firing	0.979	3743.595	2	161	<0.001
Number of firing ^∗^ block type	0.508	27.565	4	324	<0.001
Number of firing ^∗^ shade type	0.102	9.173	2	161	<0.001
Number of firing ^∗^ thickness	1.035	86.809	4	324	<0.001
Number of firing ^∗^ block type ^∗^ shade type	0.495	26.648	4	324	<0.001
Number of firing^∗^ block type ^∗^ thickness	0.498	13.444	8	324	<0.001
Number of firing ^∗^ shade type ^∗^ thickness	0.382	19.127	4	324	<0.001
Number of firing ^∗^ block type ^∗^ shade type ^∗^ thickness	0.491	13.188	8	324	<0.001

ANOVA, *p* < 0.05 indicates a significant difference at repeated measurements.

**Table 4:** Mean TP values and multiple comparison for different number of firings, block types, shade types, and sample thicknesses.

Block	Shade type	Thickness	1st firing	3rd firing	5th firing
XT	Preshaded	0.5 mm	27.63 ± 1.10^Aa^	24.86 ± 0.96^Ba^	25.74 ± 1.07^Ca^
		1 mm	21.81 ± 0.83^Ab^	19.65 ± 0.77^Bb^	20.17 ± 0.94^Bb^
		1.5 mm	17.74 ± 0.76^Ac^	15.42 ± 0.60^Bc^	16.31 ± 0.55^Cc^
	Shaded	0.5 mm	24.71 ± 2.84^Ad^	21.84 ± 0.66^Bd^	23.37 ± 0.88^Cd^
		1 mm	20.17 ± 0.77^Ab^	18.36 ± 0.64^Be^	19.44 ± 0.63^Ab^
		1.5 mm	16.58 ± 0.57^Ac^	15.40 ± 0.45^Bc^	16.68 ± 0.55^Ac^
ST	Preshaded	0.5 mm	23.37 ± 0.82^Aa^	21.48 ± 0.66^Ba^	22.64 ± 0.61^Aa^
		1 mm	18.18 ± 0.54^Ab^	17.01 ± 0.50^Bb^	19.16 ± 0.63^Cb^
		1.5 mm	14.80 ± 0.52^Ac^	13.41 ± 0.49^Bc^	13.82 ± 0.39^Bc^
	Shaded	0.5 mm	21.21 ± 0.61^Ad^	18.45 ± 0.46^Bd^	20.05 ± 0.42^Cd^
		1 mm	18.81 ± 0.60^Ab^	16.51 ± 0.34^Bb^	17.74 ± 0.37^Ce^
		1.5 mm	14.84 ± 0.52^Ac^	12.95 ± 0.53^Bc^	13.41 ± 0.32^Bc^
HT	Preshaded	0.5 mm	18.11 ± 0.40^Aa^	16.54 ± 0.44^Ba^	17.41 ± 0.37^Aa^
		1 mm	14.62 ± 0.41^Ab^	12.95 ± 0.33^Bb^	13.43 ± 0.26^Bb^
		1.5 mm	10.64 ± 0.40^Ac^	9.32 ± 0.26^Bc^	10.25 ± 0.40^Ac^
	Shaded	0.5 mm	18.50 ± 0.31^Aa^	15.91 ± 0.38^Bd^	16.72 ± 0.42^Cd^
		1 mm	13.42 ± 0.25^Ad^	11.31 ± 0.38^Be^	12.17 ± 0.47^Ce^
		1.5 mm	10.10 ± 0.46^Ae^	9.24 ± 0.45^Bc^	9.87 ± 0.28^Ac^

Average values with the same letter do not differ significantly from each other. Capital letters indicate significant differences between firing numbers (*p* < 0.05); lowercase letters indicate differences between staining and sample thicknesses (*p* < 0.05).

The article "Effect of Repeated Firings and Thickness on Optical Properties of Variable Preshaded and Shaded Novel Translucent Zirconia Blocks" was published in 2022. Journal: Biomed Res Int.

**Table 5:** Mean values of ∆*E* and multiple comparisons for number of firings, block type, shade type, and sample thicknesses.

Block	Shade type	Thickness	1-3 firings	1-5 firings	3-5 firings
XT	Preshaded	0.5 mm	3.61 ± 0.27^Aa^	5.87 ± 0.36^Bad^	5.44 ± 0.41^Ca^
		1 mm	5.12 ± 0.22^Ab^	6.16 ± 0.16^Bac^	3.28 ± 0.23^Cb^
		1.5 mm	5.94 ± 0.30^Ac^	6.90 ± 0.38^Bb^	3.51 ± 0.23^Cbc^
	Shaded	0.5 mm	3.95 ± 0.27^Aa^	6.07 ± 0.20^Bac^	5.64 ± 0.28^Ca^
		1 mm	5.35 ± 0.31^Ab^	6.41 ± 0.22^Bcd^	3.54 ± 0.29^Cbc^
		1.5 mm	6.17 ± 0.21^Ac^	7.05 ± 0.19^Bb^	3.78 ± 0.34^Cc^
ST	Preshaded	0.5 mm	2.78 ± 0.16^Aa^	4.91 ± 0.17^Ba^	4.70 ± 0.37^Ba^
		1 mm	4.62 ± 0.21^Ab^	5.11 ± 0.15^Ba^	2.72 ± 0.22^Cb^
		1.5 mm	5.18 ± 0.16^Ac^	6.26 ± 0.13^Bb^	3.11 ± 0.20^Cc^
	Shaded	0.5 mm	3.01 ± 0.27^Aa^	5.95 ± 0.32^Bc^	5.40 ± 0.20^Cd^
		1 mm	5.06 ± 0.15^Ac^	6.27 ± 0.22^Bb^	3.17 ± 0.15^Cc^
		1.5 mm	5.86 ± 0.13^Ad^	6.83 ± 0.16^Bd^	3.22 ± 0.25^Cc^
HT	Preshaded	0.5 mm	2.22 ± 0.15^Aa^	4.41 ± 0.19^Ba^	4.23 ± 0.11^Ba^
		1 mm	4.28 ± 0.12^Ab^	4.76 ± 0.15^Bb^	2.38 ± 0.15^Cb^
		1.5 mm	5.19 ± 0.17^Ac^	5.99 ± 0.16^Bc^	2.66 ± 0.11^Cc^
	Shaded	0.5 mm	2.95 ± 0.15^Ad^	4.81 ± 0.16^Bb^	4.77 ± 0.11^Bd^
		1 mm	3.88 ± 0.19^Ae^	5.19 ± 0.07^Bd^	3.99 ± 0.14^Ae^
		1.5 mm	6.70 ± 0.09^Af^	6.65 ± 0.11^Ae^	4.26 ± 0.13^Ba^

Average values with the same letter do not differ significantly from each other. Capital letters indicate significant differences between firing numbers (*p* < 0.05); lower case letters indicate the differences between shade type and sample thicknesses (*p* < 0.05).

## Data Availability

The statistical data used to support the findings of this study are available from the corresponding author upon request.
